The article "Analytical Model of Action Fusion in Sports Tennis Teaching by Convolutional Neural Networks" was published in 2022. Journal: Comput Intell Neurosci.

# Analytical Model of Action Fusion in Sports Tennis Teaching by Convolutional Neural Networks

**DOI:** 10.1155/2022/7835241

**Published:** 2022-07-31

**Authors:** Huiguang Li, Hanzhao Guo, Hong Huang

**Affiliations:** ^1^School of Education, Zhanjiang University of Science and Technology, Zhanjiang, Guangdong 524084, China; ^2^Graduate School, Guangzhou Sport University, Guangzhou, Guangdong 510500, China; ^3^School of Sports Science, Lingnan Normal University, Zhanjiang, Guangdong 524048, China

## Abstract

In order to improve the effectiveness of tennis teaching and enhance students' understanding and mastery of tennis standard movements, based on the three-dimensional (3D) convolutional neural network architecture, the problem of action recognition is deeply studied. Firstly, through OpenPose, the recognition process of human poses in tennis sports videos is discussed. Athlete tracking algorithms are designed to target players. According to the target tracking data, combined with the movement characteristics of tennis, real-time semantic analysis is used to discriminate the movement types of human key point displacement in tennis. Secondly, through 2D pose estimation of tennis players, the analysis of tennis movement types is achieved. Finally, in the tennis player action recognition, a lightweight multiscale convolutional model is proposed for tennis player action recognition. Meanwhile, a key frame segment network (KFSN) for local information fusion based on keyframes is proposed. The network improves the efficiency of the whole action video learning. Through simulation experiments on the public dataset UCF101, the proposed 3DCNN-based KFSN achieves a recognition rate of 94.8%. The average time per iteration is only 1/3 of the C3D network, and the convergence speed of the model is significantly faster. The 3DCNN-based recognition method of information fusion action discussed can effectively improve the recognition effect of tennis actions and improve students' learning and understanding of actions in the teaching process.

## 1. Introduction

Tennis is an intense and elegant sport that integrates entertainment, fitness, viewing, and competition. It is also known as “the second-largest ball game in the world” [1–3]. In the mid-19th century, tennis was introduced to China, when very few people played tennis. Today, tennis has entered the life of ordinary residents and has become one of the lifestyles advocated by modern society. Tennis has a history of hundreds of years. It has a relatively profound cultural heritage and an elegant sports tradition. This sport has a far-reaching impact on the development of today's sports world. Tennis appears in front of people with a healthy and fashionable image. Therefore, compared with other ball games, tennis is more likely to be liked by college students and other youth groups [4, 5]. In the eyes of young students, tennis can better show their style. When hitting the ball, the lower limbs push the ground hard, and as the body rotates, the upper and lower limbs are required to coordinate and cooperate in driving the arms racket to hit the ball. The large and small muscle groups of the neck, shoulders, chest, back, waist, and legs work together to complete the action.

The problem of object detection has always received much attention in the field of computer vision. Zhang et al. used the classic sliding window and image scaling to solve general object detection problems. The cost of the object detection process using this method is too high [6]. Xiao et al. proposed a fast region-convolutional neural network (Fast R-CNN) in the process of target detection and region-convolutional neural network (R-CNN) was optimized. They solved the problem that R-CNN was slow in detection [7]. Zhong et al. used the region proposal network for real-time object detection. After repeatedly using multiple regions for object detection, they found that the results of regional object detection and convolutional neural network (CNN) object detection were the same [8]. Zhao et al. used a trained object detector to detect the object at the predicted position of the next frame and updated the detector according to the detection result [9]. Ren and Han used scale pooling technology to scale the image at multiple scales and used translation filters to detect objects on it and take the corresponding maximum position and scale [10]. Elhoseny used Kalman filtering to propagate the tracked object state into future frames and associate current detections with existing objects, managing the age of tracked objects [11]. Cheng et al. introduced a pedestrian reidentification dataset in pedestrian object recognition to improve sort object tracking [12]. Ryselis et al. combined and tracked 10–12 key nodes in the human body to identify various types of actions [13]. Xie et al. used a depth camera to read human skeleton information composed of key points to estimate human pose and motion [14]. Zhang used the bottom-up idea to design some affinity field vectors to represent the skeletal orientation information of the human body, which ensures the high accuracy of human pose recognition [15]. Zhang et al. combined a novel CNN for pose regression and kinematic skeleton fitting. Two-dimensional and three-dimensional stereo techniques are used for regression and modeling of human joint position. A coherent human pose joint system based on a kinematic skeleton was established. Within a certain period, stable body posture joint information is output [16].

Under the background of the gradual diversification of physical education teaching in colleges and universities, in tennis teaching in colleges and universities, the key to correcting training movements is to accurately detect wrong movements to ensure those wrong movements are corrected in time. Tennis match videos are analyzed, mainly focusing on the sports behavior of the two major goals of athletes and tennis, to understand the key technical points and to improve the level of personal ability [17–19]. In the problem of human action recognition and processing in the video, the human pose changes continuously in time. Therefore, an action recognition method based on trajectory features is used to track the human state. In tennis match videos, the video frame occupied by the players is usually small. Therefore, in the action analysis, the algorithm needs to obtain the human skeleton information from the fine-grained analysis, and then calculate the displacement of the key points to obtain the sports data of the athlete [20–22]. Compared with traditional methods, the action recognition method based on deep learning can automatically learn relevant features from the original video and improve the action recognition rate.

At present, many mature deep learning methods have been gradually applied in the field of action recognition. Firstly, tennis players are subjected to 2D pose estimation, enabling analysis of their movement types. Next, an action recognition method based on the three-dimensional convolutional neural network (3D CNN) architecture is proposed for the needs of human action recognition in long videos. This method is combined with the key frame segment network (KFSN) based on local information fusion of keyframes to improve the efficiency of learning the whole tennis action video. The innovation point is to improve the effect of tennis sports teaching by combining the overall movements of the human body in sports tennis. It is different from the technical analysis of tennis videos under the previous deep learning method. After the tennis sports are analyzed, the teaching is carried out, and the significance of tennis sports analysis is extended, which has certain practical value. Additionally, the action recognition of the tennis sports process is further explored.

## 2. Method

### 2.1. Recognition of 2D Human Pose in Tennis Video

Tennis is a skill-dominated sport with net-separated confrontational items. Players control the tennis ball with rackets in their respective half courts to limit the opponent's performance. Compared with sports dominated by physical fitness, tennis is dominated by tactical ability. Through the analysis of tennis match videos, the technical points of professional athletes are clearly understood. This is of great help in improving personal and professional ability. Traditional computer vision methods will consider the use of depth information, such as the Kinect camera can collect depth information. Therefore, pattern recognition is used to estimate human pose. In the era of deep learning, finding out the action features of professional athletes from the perspective of computer vision is the best way to recognize action poses. In tennis sports videos, 2D human pose recognition mainly obtains skeleton information from images. That is, it needs to know the position of human joints and the connection relationship between joints [23]. The motion types of each joint of the human body belong to different channels, which are predictable outside the neural network. Therefore, the positions of each joint are connected in a predefined order to obtain a complete skeleton of a person.

OpenPose, as a two-dimensional human pose estimation algorithm using a partial affinity domain, relied on a CNN and supervised learning to achieve human pose evaluation [24–26]. Like many bottom-up methods, firstly, OpenPose detects the joints (key points) of all people in the image and assigns the detected key points to each corresponding person. Its main advantage is that it is suitable for multiperson, 2D, and more accurate identification of open-source models. A complete human image can find 18 joint points of the human body through OpenPose, as shown in Figure 1. Firstly, an image is an input, and features are extracted using a VGG19 convolutional network. VGG19 has a total of 19 layers, including 16 layers of convolution and three fully connected layers, with a pooling layer in the middle, and finally the result is output through softmax layer. Each layer of the neural network uses the output of the previous layer to extract more complex features until it is complex enough to be used to recognize images. Therefore, each layer can be regarded as an extractor of many local features, resulting in a set of feature maps. Then, a CNN network is used to extract confidence and association. Even matching in graph theory is used to find the part association. The joint points of the same person are connected. Due to the vector nature of the part affinity field (PAF) itself, the generated couples are correctly matched and finally merged into the overall skeleton of a person.

### 2.2. Real-Time Semantic Analysis of Tennis Match Videos

A set of real-time semantic intelligent analysis systems is built for the two types of sports targets, athletes, and tennis in tennis video games, as shown in Figure 2. The semantic analysis mainly designs two modules, the movement data statistics and real-time movements and the trajectory and landing prediction analysis module of tennis players [27]. From the perspective of the athlete, firstly, the target of the athlete in the video is detected. Continuous tracking after the target is locked. In this process, more nuanced categories are used to characterize athletes and provide more specific semantic information. Calculations of key point displacements are used to derive the athlete's movement data. From a tennis perspective, tennis is a smaller target in the video than the athlete. Moreover, tennis is usually in a high-speed running state when it is in motion. Therefore, in some video frames, the movement of the tennis ball is almost indistinguishable to the naked eye. In the process of semantic analysis of tennis balls, firstly, motion vectors are obtained from nonconsecutive video frames that can be detected. Combined with the motion characteristics of tennis balls (oblique throwing motion), the prediction of the landing area of tennis balls is realized.

In Figure 2, the surveillance camera is responsible for capturing video of tennis games. The server is responsible for preprocessing the video, including handling its format, exposure, and noise. The processed video data is transmitted to the client through socket communication. The client acts as a bridge between the server and the user, and displays the processing results to the user. Second, semantic analysis is used to map the visual and semantic features of tennis sports videos into a common embedding space to address the semantic inconsistency between video content and generated descriptions. Semantic consistency is achieved by minimizing the Euclidean distance between two embedded features. After semantic analysis, the movement data of tennis players are obtained. The tennis ball landing area is predicted. In order to obtain the sports information of the athlete through analysis, the algorithm flow of the real-time semantic parsing of the adopted sportsman's sports is shown in Figure 3. In the semantic parsing algorithm, firstly, the input high-definition tennis match video is subjected to object detection, that is, players and tennis balls are detected [28, 29]. Then, different athletes are identified and the target athlete is identified and continuously tracked. Next, the skeletal key points of the target athlete are detected. The acquired position information of each key point is used to complete the discrimination of the athlete's action, that is, to output the semantic information. The channel feature fusion algorithm obtains the visual saliency map of multiuser-generated videos. These videos are mapped into the manifold. Finally, multiple attributes are used to extract keyframes from multiple videos.

### 2.3. Action Recognition Based on 3D Lightweight Multiscale CNN

In the early days, a classic attempt to apply deep learning to RGB video was to extend 2D CNN to form a two-stream architecture to obtain spatial features of video frames and motion features between frames, respectively [30–32]. An image is a projection from real-world 3D coordinates to 2D plane coordinates. Therefore, a straightforward method for 3D object detection from an image is to inverse transform the 2D image to 3D world coordinates and perform object detection in the world coordinate system. The video itself has more 3D volumes in the temporal dimension. The 3D network intuitively uses the 3D convolution kernel to obtain the spatiotemporal features of the video by means of the regularization of high-level features. With this structure, the feature maps in the convolutional layer are all connected to multiple adjacent frames in the previous layer, capturing motion information. The time dimension is taken as the 3D, and 3D convolution is formed by stacking multiple consecutive frames to form a cube. Then, a 3D convolution kernel is applied to the cube. In this structure, each feature map in the convolutional layer is connected to multiple adjacent consecutive frames in the previous layer to capture motion information. The 3D convolution kernel extracts one type of feature from the cube. During the entire convolution process, the weights of the convolution kernels are the same (shared weights), which are the same convolution kernel. The convolution process of the 3D CNN model is shown in Figure 4. Only 3D convolution preserves the temporal information of the input signal, resulting in the output volume. The same phenomenon also applies to 2D and 3D pooling. Although the temporal flow network takes multiple frames as input, the temporal information completely disappears due to the 2D convolution after the first convolutional layer. Fusion models use 2D convolutions, and most networks lose the temporal signal of their inputs after the first convolutional layer.

The 3D convolution is shown in the following equations:

(1) $$\begin{array}{c} F^{\prime }=F*K, \end{array}$$

(2) $$\begin{array}{c} F_{j}^{\prime xyz}=\sum_{n}\sum_{h=0}^{h_{k}-1}\sum_{w=0}^{w_{k}-1}\sum_{t=0}^{t_{k}-1}K_{jn}^{hwt}F_{n}^{\left(x+h\right)\left(y+w\right)\left(z+t\right)}. \end{array}$$

Here, *F*′ represents the intermediate feature map, *K* represents the 3D convolution kernel, *F*_*j*_^′*xyz*^ represents the value of the *j*-th feature map at the (*x*, *y*, *z*) spatial position, *K*_*jn*_^*hwt*^ represents the *j*-th convolution kernel connected to the *n*-th feature map at the spatial coordinate (*x*, *y*, *z*) value, *t* represents the length of the time domain, and *hw* represent the height and width of the airspace, respectively.

The input to the 3D CNN model is restricted to a few consecutive video frames. As the size of the input window increases, the parameters that the model needs to train also increase. Therefore, in the 3D CNN model, such high-level motion information is captured. Many frames are used to compute motion features. These motion features are then used as auxiliary outputs to regularize the 3D CNN model. For each behavior that needs to be trained, its long-term behavior information is extracted as its high-level behavior features. The last hidden layer of the CNN is used to connect a series of auxiliary output nodes. Then, during the training process, the extracted features are closer to the calculated high-level behavioral motion feature vector.

Conventional CNN inference requires a large amount of computation and is difficult to apply in resource-constrained scenarios such as mobile terminals and the Internet of Things. Only through complex cropping and quantization CNN can be barely deployed to the mobile terminal. Starting from SqueezeNet and MobileNet v1, the design of CNN began to focus on efficiency issues in resource-constrained scenarios [33, 34]. Compared with the two-stream method, 3D CNN can directly learn spatiotemporal features from raw RGB videos. However, 3D CNN has high complexity, computational complexity, and a large memory footprint. These shortcomings impact the depth of the network, and more abstract features cannot be obtained. Therefore, a lightweight multiscale 3D CNN model is further proposed. A lightweight multiscale convolution module is embedded in the 3D residual to increase the receptive field of each layer. Based on the RetinaNet framework, a lightweight CNN is used as the backbone network to extract image features. The downsampling module is used to downsample the output multiscale feature maps. In the original RetinaNet framework, the largest-scale feature maps with the lowest proportion of detection targets are removed. The 1 × 1 convolution can change the number of channels without changing the spatial resolution of the feature maps, keeping the computational efficiency high even with a low amount of parameters. At present, the efficiency of the 1 × 1 convolution operation is supported by many underlying algorithms, which are more efficient.

### 2.4. Identification of Segmented Competition Video Based on Local Information Fusion

Each video is an image sequence, and its content is much richer than an image, with strong expressiveness and a large amount of information. Analysis of video is usually based on video frames. However, there is usually a lot of redundancy in video frames, and there are also missing frames and redundancy in its extraction. Complex athletic movements often involve multiple phases of movement over a longer period of time. Failure to use long-term temporal structures in CNN will result in a certain information loss for action recognition tasks. The keyframe extraction of video mainly reflects the salient features of each shot in the video, which can effectively reduce the time required for video retrieval and enhance the accuracy of video retrieval [35, 36]. In the video keyframe extraction method based on deep learning, the extraction efficiency of keyframes can be greatly improved without mastering various features of video images. The keyframe detection network AdaScan is used to complete the extraction of keyframes from tennis match videos. After AdaScan receives the features of each frame of the video, its importance for recognition is determined and aggregated into a deep learning framework. The extraction process of the key frame detection network AdaScan is shown in Figure 5.

In Figure 5, firstly, a hierarchical clustering algorithm is used to extract video keyframes initially. Then, combined with the semantic correlation algorithm, the preliminarily extracted keyframes are compared by histograms to remove redundant frames. The keyframes of the video are determined. In order to apply long-term temporal structure to CNN training, KFSN based on local information fusion is proposed to achieve long-term dynamic modeling of the entire video [37]. Firstly, a video *V* is given. It is divided into *K* equally spaced paragraphs {*S*_1_, *S*_2_ … *S*_*k*_}. Then, KFSN models the sequence of video clips as shown in the following equation:

(3) $$\begin{array}{c} \text{KFSN}\left(F_{1},F_{2}\ldots F_{k}\right)=H\left(T\left(f\left(F_{1};W\right),f\left(F_{2};W\right)\ldots f\left(F_{k};W\right)\right)\right). \end{array}$$

Here, (*F*_1_, *F*_2_ … *F*_*k*_) denotes a video frame sequence, *F*_*k*_ is a keyframe, and *H* denotes a prediction function.

The final loss function of the piecewise consistency function is obtained, as shown in the following equation:

(4) $$\begin{array}{c} L\left(y,G\right)=-\sum_{i=1}^{c}y_{i}\left(G_{i}-\log\sum_{j=1}^{c}\exp\;G_{i}\right). \end{array}$$

Here, *c* denotes the number of action classes, *y*_*i*_ denotes the ground-truth labels associated with the action class, and *G* denotes the consensus function.

The video fixation of the same experiment is uniformly divided into K segments. Each video is sparsely sampled based on temporal length. Only a few frames are covered in the video, and they are all keyframes. A two-stream network structure is adopted, and a fixed number of frames (25 frames) are sampled in the action video. The weight of the spatial stream is set to 1, and the weight of the temporal stream is set to 1.5.

### 2.5. Experimental Setup

The public dataset UCF101 is chosen to validate the performance of the proposed 3D CNN-based KFSN model. UCF101 is an action recognition dataset for realistic action videos, collected from YouTube, providing 13320 videos from 101 action categories. The sample distribution of the UCF101 dataset is shown in Table 1. Videos with a video length greater than 20 seconds are selected as test samples. Videos of 10–20 seconds are used as training samples, keeping the ratio of the two at 8 : 2. There are two ways to process and load data: generate a PKL file from the video file for processing or directly process the video. The designed KFSN model covers a 35-layer network, two pooling layers and two fully connected layers, 30 convolutional layers, and a dropout. The convolution kernel size of the first convolutional layer is set to 7 × 7, and the convolution kernel sizes of the remaining layers are 1 × 1 and 3 × 3.

The processor of this experiment is Intel i7 2.6 GHz and the operating system is Ubuntu 16.04. The specific information on hyperparameter configuration is shown in Table 2. RGB image keyframe and optical flow map are taken as input, and the method of spatial + temporal training is adopted for processing.

## 3. Results and Discussion

### 3.1. Evaluation of the Performance of the Semantic Analysis System for Tennis Match Videos

In order to accurately evaluate the accuracy of the server-side algorithm, three groups of experiments are conducted separately. Three groups of experiments provide data comparison when performing performance analysis of the semantic analysis system of tennis game videos. The same system is used to discriminate the athlete's movement type accurately. The difference is that different discriminative effects of the action of the target athlete can be displayed. A video is randomly selected from the four-game scenarios in the database. Compare the difference between the output value of the semantic analysis algorithm and the real value to evaluate the discriminative effect of the target athlete's action.  Figure 6 is the experimental result of the video semantic analysis system to discriminate the type of athlete's action. The scene has little effect on the accuracy of the system's action discrimination. In the three groups of experiments, the system's accuracy for judging athlete movements is maintained between 50% and 100%. The discriminative accuracy of the proposed semantic analysis system for athlete swings is low in each scene. The reason may be that the target athlete has his back to the camera during the game. Therefore, in some video frames, the key points on the arm are severely occluded, which affects the recognition of the swing by the system.

### 3.2. Action Recognition Rate of KFSN Model Based on 3D CNN

After 16 iterations of the model, UCF101 achieves 91.4% accuracy for action recognition. Compared with the traditional 3D CNNC3D, the evaluation indicators include model complexity and training time, as shown in Figure 7. The structure of C3D is relatively simple, and the model covers eight convolutional layers, five pooling layers, two fully connected layers, and a Softmax classification layer. Compared with the entered KFSN model, the convolution kernel size of all convolutional layers in C3D is fixed, which is 3 × 3 × 3. The number of neurons in each fully connected layer is 4096. The proposed 3D CNN-based KFSN model is only 1/3 of the C3D model's average iteration time. The model speeds up convergence while ensuring recognition accuracy.

## 4. Conclusion

Currently, video analytics and the entire technology stack of big data systems rely on deep learning. Video content analysis requires a relatively complete understanding of the video content and applying it to the analysis of sports events can more accurately understand the movement skills of athletes. This is very important for the teaching of special sports. The traditional action recognition method cannot accurately obtain the wrong action characteristics of physical education training, which affects the detection accuracy. As a result, the quality of special education is reduced. Deep learning methods have been successfully applied in object tracking and gradually surpassed traditional methods in performance. Firstly, the design and implementation of a real-time semantic analysis system for tennis match videos are introduced. In the specific game video analysis, the video itself has a 3D volume in the time dimension. Many frames are used to compute motion features. These motion features are then used as auxiliary outputs to regularize the 3D CNN model. In addition, a 3DCNN-based KFSN model based on local information fusion is proposed. The model implements long-term dynamic modeling of the entire video. Finally, the performance of the proposed model is verified on the public dataset UCF101. The model achieved an accuracy of 91.4% for action recognition. Compared with the C3D model, the average iteration time is only 1/3 of the C3D model. The designed action analysis model for sports tennis teaching based on CNN has a good realization in terms of accuracy and stability. The target recognition model based on the neural network can realize the skill analysis of tennis game videos, which greatly value tennis teaching. However, the discussed semantic analysis fails to consider the interaction between people and objects in actual scenes. The action discrimination involved is relatively simple, and further breakthroughs are needed to recognize and analyze complex interactive actions.

## Figures and Tables

**Figure 1:** Schematic representation of human joint points.

**Figure 2:** Architecture of a real-time semantic analysis system for tennis match videos.

**Figure 3:** Flow of the parsing algorithm for motion real-time semantics.

**Figure 4:** Convolution process of the 3D CNN model.

**Figure 5:** Extraction process of keyframe detection network AdaScan.

**Figure 6:** The results of the video semantic analysis system discriminating the type of athlete's action.

**Figure 7:** Comparison of the proposed model with C3D.

**Table 1:** Situation of the sample distribution of the UCF101 dataset.

Dataset	Classes	Videos		Clips	
		Train	Test	Train	Test
UCF101	101	10656	2664	10656	2664

**Table 2:** Configuration information of neural network hyperparameters.

Convolution type	Parameter index	Value
Temporal convolution	Batch size	256
	weight_decay	5 × 10^−4^
	max_iter	2000
	Site value	[1200, 1800]
	Momentum	0.8

Spatial convolution	Batch size	256
	weight_decay	5 × 10^−4^
	max_iter	4300
	Stepsize	2000
	Momentum	0.8

## Data Availability

The dataset used in this paper are available from the corresponding author upon request.

## References

[1] Kilit B., Arslan E., Soylu Y. (2018). Time-motion characteristics, notational analysis and physiological demands of tennis match play: a review. *Acta Kinesiologica*.

[2] González-García H., Martinent G. (2020). Relationships between perceived coach leadership, athletes’ use of coping and emotions among competitive table tennis players. *European Journal of Sport Science*.

[3] Swettenham L., Eubank M., Won D., Whitehead A. E. (2020). Investigating stress and coping during practice and competition in tennis using think aloud. *International Journal of Sport and Exercise Psychology*.

[4] Tsuda E., Ward P., Goodway J. D. (2018). Defining tennis content in upper elementary physical education. *Journal of Physical Education, Recreation and Dance*.

[5] Biernat E., Buchholtz S., Krzepota J. (2018). Eye on the ball: table tennis as a pro-health form of leisure-time physical activity. *International Journal of Environmental Research and Public Health*.

[6] Zhang Y., Yuan Y., Feng Y., Lu X. (2019). Hierarchical and robust convolutional neural network for very high-resolution remote sensing object detection. *IEEE Transactions on Geoscience and Remote Sensing*.

[7] Xiao Y., Wang X., Zhang P., Meng F., Shao F. (2020). Object detection based on faster R-CNN algorithm with skip pooling and fusion of contextual information. *Sensors*.

[8] Zhong Z., Sun L., Huo Q. (2019). An anchor-free region proposal network for Faster R-CNN-based text detection approaches. *International Journal on Document Analysis and Recognition*.

[9] Zhao X., Sun P., Xu Z., Min H., Yu H. (2020). Fusion of 3D LIDAR and camera data for object detection in autonomous vehicle applications. *IEEE Sensors Journal*.

[10] Ren J., Han J. (2021). A new multi-scale pedestrian detection algorithm in traffic environment. *Journal of Electrical Engineering & Technology*.

[11] Elhoseny M. (2020). Multi-object detection and tracking (MODT) machine learning model for real-time video surveillance systems. *Circuits, Systems, and Signal Processing*.

[12] Cheng K., Tao F., Zhan Y., Li M., Li K. (2020). Hierarchical attributes learning for pedestrian re-identification via parallel stochastic gradient descent combined with momentum correction and adaptive learning rate. *Neural Computing & Applications*.

[13] Ryselis K., Petkus T., Blažauskas T., Maskeliūnas R., Damaševičius R. (2020). Multiple Kinect based system to monitor and analyze key performance indicators of physical training. *Human-Centric Computing and Information Sciences*.

[14] Xie P., Liang X., Song Y., Cai Z. (2020). Mass spectrometry imaging combined with metabolomics revealing the proliferative effect of environmental pollutants on multicellular tumor spheroids. *Analytical Chemistry*.

[15] Zhang R. (2022). Analyzing body changes of high-level dance movements through biological image visualization technology by convolutional neural network. *The Journal of Supercomputing*.

[16] Zhang D., Wu Y., Guo M., Chen Y. (2021). Deep learning methods for 3D human pose estimation under different supervision paradigms: a survey. *Electronics*.

[17] Kocib T., Carboch J., Cabela M., Kresta J. (2020). Tactics in tennis doubles: analysis of the formations used by the serving and receiving teams. *Int J Phys Educ Fit Sport*.

[18] Jiang W., He G. (2021). Study on the effect of shoulder training on the mechanics of tennis serve speed through video analysis. *Molecular & Cellular Biomechanics*.

[19] Ellis D. G., Speakman J., Hambly C. (2021). Energy expenditure of a male and female tennis player during association of tennis professionals/women’s tennis association and grand slam events measured by doubly labeled water. *Medicine & Science in Sports & Exercise*.

[20] Zhang H., Zhou Z., Yang Q. (2018). Match analyses of table tennis in China: a systematic review. *Journal of Sports Sciences*.

[21] Zhou Q., Zhong B., Lan X. (2020). Fine-grained spatial alignment model for person re-identification with focal triplet loss. *IEEE Transactions on Image Processing*.

[22] Ma M., Marturi N., Li Y., Leonardis A., Stolkin R. (2018). Region-sequence based six-stream CNN features for general and fine-grained human action recognition in videos. *Pattern Recognition*.

[23] Wan C., Wu Y., Tian X., Huang J., Hua X. -S. (2019). Concentrated local part discovery with fine-grained part representation for person re-identification. *IEEE Transactions on Multimedia*.

[24] Nadeem A., Jalal A., Kim K. (2021). Automatic human posture estimation for sport activity recognition with robust body parts detection and entropy Markov model. *Multimedia Tools and Applications*.

[25] Wu E. Q., Tang Z. R., Xiong P., Wei C. -F., Song A., Zhu L. -M. (2021). ROpenPose: a rapider OpenPose model for astronaut operation attitude detection. *IEEE Transactions on Industrial Electronics*.

[26] Jo B. J., Kim S. K. (2022). Comparative analysis of OpenPose, PoseNet, and MoveNet models for pose estimation in mobile devices. *Traitement du Signal*.

[27] Lin C. B., Dong Z., Kuan W. K., Huang Y.-F. (2020). A framework for fall detection based on OpenPose skeleton and LSTM/GRU models. *Applied Sciences*.

[28] Farhat M., Khalfallah A., Bouhlel M. S. (2018). A new model based approach for tennis court tracking in real time. *International Journal of Signal and Imaging Systems Engineering*.

[29] Peng X., Tang L. (2022). Biomechanics analysis of real-time tennis batting images using Internet of Things and deep learning. *The Journal of Supercomputing*.

[30] Gu D. (2018). Analysis of tactical information collection in sports competition based on the intelligent prompt automatic completion algorithm. *Journal of Intelligent and Fuzzy Systems*.

[31] Gong H., Li Q., Li C. (2021). Multi-scale information fusion for hyperspectral image classification based on hybrid 2D-3D CNN. *Remote Sensing*.

[32] Xu Q., Xiao Y., Wang D., Luo B. (2020). CSA-MSO3DCNN: multi-scale octave 3D CNN with channel and spatial attention for hyperspectral image classification. *Remote Sensing*.

[33] Ghadai S., Lee X. Y., Balu A., Sarkar S., Krishnamurthy A. (2021). Multi-resolution 3D CNN for learning multi-scale spatial features in CAD models. *Computer Aided Geometric Design*.

[34] Wang J., Huang R., Guo S. (2021). NAS-guided lightweight multi-scale attention fusion network for hyperspectral image classification. *IEEE Transactions on Geoscience and Remote Sensing*.

[35] Li J., Zhang S., Huang T. (2020). Multi-scale temporal cues learning for video person re-identification. *IEEE Transactions on Image Processing*.

[36] Mademlis I., Tefas A., Pitas I. (2018). A salient dictionary learning framework for activity video summarization via keyframe extraction. *Information Sciences*.

[37] Xiao-Gen P. (2021). The key frame extraction algorithm based on the indigenous disturbance variation difference video. *Procedia Computer Science*.

